The article "Curcumin Inhibits the Proliferation of Renal Cancer 786-O Cells through MTOR Signaling Pathway and Its Mechanism" was retracted in 2023. Reasons: suspected computer-generated content; unreliable results or conclusions; concerns about the data; concerns about the results or conclusions.

# Curcumin Inhibits the Proliferation of Renal Cancer 786-O Cells through MTOR Signaling Pathway and Its Mechanism

**DOI:** 10.1155/2022/1842389

**Published:** 2022-03-30

**Authors:** Rui Gao, Yunfang Ma, Yali Wang, Haili Xu

**Affiliations:** ^1^Department of Oncology, Jinan Municipal Hospital of Traditonal Chinese Medicine, Jinan 250012, China; ^2^Disinfection and Supply Center, East Hospital, Qingdao Municipal Hospital, Qingdao 266000, China; ^3^Comprehensive Oncology Department, The Affiliated Qingdao Central Hospital of Qingdao University, The Second Affiliated Hospital of Medical College of Qingdao University, Qingdao 266042, China

## Abstract

**Objectives:**

The mechanism of curcumin inhibiting renal cancer 786-O cells proliferation through MTOR signaling pathway was investigated.

**Methods:**

Human renal cancer 786-O cells were cultured with curcumin for 48 h. The OD values were measured by the MTT method, and the growth inhibition rate of 786-O cells was calculated. The cell cycle distribution and apoptosis rate were detected by flow cytometry (FCM). Transwell chamber was introduced to detect cell invasion ability. Cell migration ability was detected by the cell scratch test. The protein expression was assessed by Western blot.

**Results:**

With curcumin concentration increasing, the expressions of MMP2, MMP9, MTOR, and p-MTOR proteins and the number of cells in the S phase decreased gradually, while number of cells in G1 and G2/M phases and cells apoptosis rate increased continuously. With the increasing of concentration and time, growth of 786-O cells in each treatment group was inhibited to varying degrees. The higher the inhibition rate was, the cells migration and transmembrane cells proportion decreased significantly.

**Conclusions:**

Curcumin inhibits the proliferation, migration, and invasion and induces apoptosis of renal cancer 786-O cells by blocking the MTOR signaling pathway. It may be related to the downregulation of MMP2 and MMP9 proteins.

## 1. Introduction

Renal cancer which originates from renal parenchymal urinary tubule epithelial cells, accounts for about 2%∼3% of adult malignant tumors [1]. Because renal cancer is not sensitive to chemotherapy, radiotherapy, and hormone therapy, its main treatment is surgery [2]. However, 20%∼40% of patients have recurrence and metastasis, and the prognosis is poor [3]. Therefore, it is necessary to explore a new treatment. Curcumin is a natural phenolic pigment extracted from the roots of radix curcuma, curcuma zedoaria, curcuma aromatica, and acori tatarinowii rhizoma [4]. Studies have found that curcumin has various pharmacological effects, such as lowering blood lipids, anti-inflammatory [5], antioxidant [6], anticoagulant, analgesic [7], antiviral [8], antiatherosclerosis, antitumor [9], and antimutation. Curcumin with spleen and liver-meridian is often used for postoperative pain, amenorrhea, rheumatism shoulder, and arm pain [10, 11]. In particular, it has the advantages of broad spectrum anticancer, small toxic and side effects, and can inhibit the growth many tumor cells in vitro. In recent years, curcumin has been reported to hamper cells growth of liver cancer [12], stomach cancer [13], lung cancer [14],and other tumor, and has the effect of inhibiting tumor progression. In vitro experiments suggested that curcumin can inhibit various tumor cells proliferation and metastasis, including colon cancer [15], prostate cancer [16], and breast cancer [17] and induce tumor cells apoptosis. At present, anticancer mechanism of curcumin needs to be improved, and its effect on human renal cancer cell lines is rarely studied.

Tumor invasion and metastasis affect patient prognosis, and inhibition of tumor invasion and metastasis is an important target for tumor treatment. MTOR signaling pathway widely exists in many cells and can participate in cell behavior, angiogenesis, and other biological characteristics by changing the activation state of downstream signal molecules [18]. In recent years, the activation of MTOR signaling pathway is related to the occurrence of various malignant tumors. It has become a new idea for cancer treatment to block the activation of downstream signaling molecules by using signaling pathway blockers to inhibit cancer cells growth [19–21]. In this study, curcumin was used to explore the effect and the possible molecular mechanism on proliferation, migration, invasion, and apoptosis of 786-O cell by blocking MTOR signaling pathway, thus providing theoretical basis for clinical drug treatment of renal cancer.

## 2. Materials and Methods

### 2.1. Cell Lines and Drugs

Cell line renal cancer cell line 786-O was purchased from Shanghai Institute of Cell Science, Chinese Academy of Sciences. Curcumin was purchased from Chengdu Sikehua Biotechnology Co., Ltd.

### 2.2. Cell Culture

Human renal cancer cell 786-O cells were applied to RPMI-1640 medium (Gibco, USA) containing 10% fetal bovine serum (FBS) (Hyclone, USA), penicillin/streptomycin, and cultured with 37°C, 5% CO_2_ incubator (Sanyo, Japan) for routine incubation. Passage was performed once every 3 days.

### 2.3. MTT Method Detection

786-O cells were digested by routine trypsin and inoculated into 96-well plates with 5 × 10^4^ cells/well. After culturing for 24 hours, 180 *μ*L of curcumin culture medium (6.25 *μ*mol/L, 12.5 *μ*mol/L, 25 *μ*mol/L, and 50 *μ*mol/L) was added. At the same time, the blank control group was added with 0 *μ*mol/L curcumin culture solution. Five replicate wells in each group were set up to continue cultivation for 24, 48, and 72 h. 20 *μ*L MTT reagent (Promega, USA) was added to each well and cells were cultured for 4 h. Each well was added with 150 *μ*L DMSO. Absorbance (OD_490_) was detected by using a microplate reader (Thermo Fisher, USA). The tumor cell inhibition rate formula is calculated as follows: cell inhibition rate = 1 − (curcumin_averageODvalue_/control_averageODvalue_) × 100%.

### 2.4. Flow Cytometry Assay

786-O cells were inoculated in 25 mL culture flask at 5 × 10^5^ cells/mL. After 24 h, cells were cultured with the medium containing different concentrations of curcumin. The cells were collected after 48 h culture and centrifuged with PBS buffer (1500 r/min, 5 min). After washing for 2 times, cells were fixed with 70% ethanol and digested with RNase enzyme. Cells were stained with 1 mL propidium bromide (PI) in a refrigerator at 4°C for 30 min and filtered with a flow cytometer (BeekmanCouher, USA). The distribution of cell cycle and apoptosis rate were calculated by using a computer software. Proliferation index (PI) was calculated according to the formula: PI = (*S* + *G*2/*M*)/(*G*0/*G*1 + *S* + *G*2/*M*).

### 2.5. Transwell Chamber Detects Cell Invasion Ability

Cell invasion ability was detected by using Transwell chambers (Corning, USA). 786-O cells were treated with curcumin medium with different concentration for 48h. The cells were digested with 0.25% trypsin. After washing with PBS, the supernatant was removed by centrifugation. The cells were then suspended in RPMI-1640 medium with 10% FBS, and cell concentration was adjusted to 1 × 10^6^ cells/mL. 100 *μ*L/well was added to the upper chamber, and 500 *μ*L RPMI-1640 medium containing 10% FBS was added to lower chamber. After incubated for 24 h, 48 h and 72 h at 37°C, the cell was fixed with methanol and stained with crystal violet. Five fields were randomly selected for observation under a microscope (Olympus, Japan).

### 2.6. Wound Healing Assay

786-O cells were inoculated into 6-well plates with 2 × 10^6^ cells/well. When degree of cell fusion >80%, a fine vertical mark was gently drawn with a pipette gun. After incubation for 24 h, 48 h, and 72 h, cell scratches width was observed with a microscope (Olympus, Japan). Five fields were randomly observed in each group to calculate cell mobility. Cell mobility = curcumin _averagewidth_/control _averagewidth_ × 100%.

### 2.7. Western Blot Assay

786-O were treated with different curcumin concentrations and digested with trypsin. The protein was extracted and measured the total concentration. The samples were quantitatively loaded for SDS-PAGE (Baygene, USA) separation. The proteins on the gel were wet-transferred onto nitrocellulose membrane at 4°C and sealed at room temperature for 60 min. After washing, membrane was incubated with primary antibody (Zhongshan Jinqiao Biotechnology Company, Beijing) for 12 h at 4°C. After washing, membrane was incubated with secondary antibody for 2 h. After the membrane was washed again for 3 times with TBS, chemiluminescence reagent (Pierce, USA) was added to develop color and exposure. Protein chemiluminescence gel imaging system (Protein Simple, USA) was used to collect images and analyze protein expression level.

### 2.8. Statistical Methods

The experimental data are expressed as $\left(\bar{x}\pm s\right)$, and the SPSS21.0 statistical software is used to perform ANOVA. *P* *<* 0.05 was considered statistically significant.

## 3. Results

### 3.1. MMP2, MMP9, MTOR, and p-MTOR Protein Expressions

The expression of MMP2, MMP9, MTOR, and p-MTOR protein in renal cancer 786-O cells treated with different curcumin concentrations was decreased versus control group (Figure 1). With increase of the dose concentration, MMP2, MMP9, MTOR, and p-MTOR protein expressions gradually decreased (Figure 1).

### 3.2. Effects of Different Curcumin Concentrations on the Growth of Renal Cancer Cell 786-O

786-O cells of the control group increased with the extension of culture time. After treatment with different curcumin concentrations, 786-O cells growth in each group was inhibited in different degrees (Figure 2). With the increase of drug concentration and culture time, the inhibition rate of 786-O cell growth was more obvious (Figure 3).

### 3.3. Effects of Different Curcumin Concentrations on Cell Cycle and Apoptosis

The distribution of cell cycle was *G*1, *S*, and *G*2/*M* peak pattern. Compared with the control group, *G*1 and *G*2/*M* phase cell number and cell apoptosis rate increased, while the cell number in the S phase decreased with the drug concentration increasing (Figures 4 and 5).

### 3.4. Effects of Different Curcumin Concentrations on Migration of 786-O Cells

The cell migration rate and cell migration distance in the control group increased with culture time extension (Table 1). Rate and distance of cell migration in other groups decreased significantly with concentration and culture time increasing (Table 1).

### 3.5. Effects of Different Concentrations of Curcumin on Invasion Ability of 786-O Cells

Transmembrane cells proportion in the control group increased gradually with time (Table 2). The proportion of transmembrane cells in other administration groups decreased significantly with time prolongation and increasing drug concentration (Table 2).

## 4. Discussion

Curcumin is a plant polyphenol extracted from the rhizome turmeric of the Zingiberaceae plant [4]. Curcumin can inhibit many tumors cell growth, this effect is reflected in the various stages of tumor development and invasion to other tissues [12, 13, 15, 16]. Curcumin inhibits cancer cell proliferation and induces apoptosis through multiple pathways and regulation of various tumor-related factors in vitro [22–24]. Recently, the mechanism of curcumin inhibiting tumor progression has become a research hotspot. Curcumin was confirmed to significantly inhibit proliferation and metastasis of breast cancer [17], liver cancer [12], prostate cancer [16], ovarian cancer [25], and a series of tumors. Beevers et al. found that curcumin can rapidly inhibit the phosphorylation of mammalian mTOR and its downstream effector molecules S6K1 and 4EBP1 in Rh1, Rh30, and other tumor cells at a physiological concentration of 2.5 *µ*m [26]. However, few research studies of curcumin have been conducted on renal cancer. Therefore, different concentrations of curcumin were used to treat renal cancer cells in this study, aiming to explore the inhibiting mechanism of curcumin inhibition on renal cancer 786-O cell proliferation through MTOR signaling pathway.

The abnormal regulation of cell proliferation and apoptosis is an important biological characteristic of malignant tumor occurrence and development. Induction of tumor cell apoptosis is an active programmed cell suicide phenomenon. Apoptosis is the key link of body balance maintenance and is closely related to tumor [27]. Experimental results showed that curcumin inhibited tumor cells proliferation and promote apoptosis [15–17]. The results suggested curcumin inhibited the growth, proliferation, and apoptosis of 786-O cells in a time-dose-dependent and dose-response manner. Loss of cell cycle is one of the important factors in the pathogenesis of tumor. If regulation of *G*1/*S* arrest points in normal cell cycle is lost, cells with damaged genomes do not undergo *G*1 arrest, resulting in uncontrolled cell proliferation and ultimately tumor formation [28]. In this study, curcumin could regulate *G*1/*S* arrest points in 786-O cells cycle and induce *G*1/*M* arrest at the same time, thereby inhibiting tumor growth and inducing apoptosis of tumor cells. Tumor cells invasion and metastasis are related to prognosis and are also the main reasons for cancer treatment failure [29]. Wound healing and Transwell chamber assay showed that curcumin inhibited the 786-O cells migration and invasion. With curcumin concentration increasing, transmembrane cells proportion, migration distance, and cell migration rate decreased gradually with a dose-dependent effect. Meanwhile, curcumin could down-regulate the expressions of MMP2, MMP9, mTOR, and P-MTOR in 786-O cells in a dose-response manner. Therefore, we speculated that curcumin may regulate the malignant behavior of 786-O cells via inhibiting the MTOR signaling pathway, indicating that curcumin has the potential of targeted drug for renal cancer treatment. However, more experiments should be performed to further confirm the effect of curcumin on two or more renal cancer cells, such as EDU experiment, apoptotic-related proteins expressions, and animal experiments.

## 5. Conclusions

As a plant-derived drug, curcumin has a low price, small toxic and side effects, and great development potential. It can inhibit the invasion and metastasis of renal cancer cells and is expected to be applied to the treatment of human cancer and chemoprophylaxis to benefit human beings.

## Figures and Tables

**Figure 1:** Protein expression (MMP2, MMP9, MTOR, and p-MTOR) of renal cell carcinoma 786-O cells under different concentrations of curcumin. ^*∗*^*P* *<* 0.05, ^*∗∗*^*P* *<* 0.01, compared with the control group.

**Figure 2:** Effect of curcumin on 786-O cell proliferation.

**Figure 3:** Inhibition rate of curcumin in different concentrations on 786-O cells.

**Figure 4:** Effect of curcumin concentration on 786-O cell cycle.

**Figure 5:** Effect of curcumin concentration on the apoptosis rate of renal cancer 786-O cells.

**Table 1:** Effect of curcumin concentration on migration of 786-O cells$\left(\bar{x}\pm s\right)$.

Curcumin concentration (*μ*mol/L)	Culture time (h)	Cell migration rate (%)	Cell migration distance (*μ*m)
0 (*n* = 5)	24	83.63 ± 1.21	256.16 ± 5.43
	48	94.67 ± 5.26	263.74 ± 5.84
	72	97.43 ± 5.74	274.87 ± 6.28
6.25 (*n* = 5)	24	89.85 ± 4.25	259.43 ± 5.74
	48	85.72 ± 4.76	245.38 ± 5.29
	72	77.76 ± 4.08	228.82 ± 5.63
12 (*n* = 5)	24	79.38 ± 3.75	213.96 ± 4.71
	48	73.68 ± 3.51	194.25 ± 4.63
	72	66.54 ± 3.26	172.66 ± 4.57
25 (*n* = 5)	24	67.31 ± 3.64	159.64 ± 4.76
	48	58.52 ± 4.67	137.82 ± 4.75
	72	48.06 ± 4.13	111.49 ± 4.38
50 (*n* = 5)	24	49.33 ± 4.58	92.36 ± 4.05
	48	40.66 ± 4.15	67.91 ± 3.18
	72	29.67 ± 3.49	42.64 ± 3.59

**Table 2:** Effect of different curcumin concentrations on the proportion of 786-O transmembrane cells$\left(\bar{x}\pm s\right)$.

Curcumin concentration (*μ*mol/L)	24 h	48 h	72 h
0 (*n* = 5)	452.46 ± 36.16	467.58 ± 35.84	486.37 ± 34.23
6.25 (*n* = 5)	431.62 ± 31.28	394.61 ± 27.42	411.37 ± 32.48
12.5 (*n* = 5)	356.83 ± 26.71	326.49 ± 18.73	334.29 ± 26.43
25 (*n* = 5)	261.76 ± 15.23	234.86 ± 14.36	274.85 ± 17.49
50 (*n* = 5)	163.48 ± 13.64	146.56 ± 11.84	102.75 ± 10.88

## Data Availability

The datasets used and/or analyzed during the present study are available from the corresponding author upon reasonable request.
